RETRACTED

# Circular RNA circ-FoxO3 Inhibits Myoblast Cells Differentiation

**DOI:** 10.3390/cells8060616

**Published:** 2019-06-19

**Authors:** Xiaoyue Li, Cunyuan Li, Zhijin Liu, Wei Ni, Rui Yao, Yueren Xu, Renzhe Quan, Mengdan Zhang, Huixiang Li, Li Liu, Shengwei Hu

**Affiliations:** 1 College of Life Sciences, Shihezi University, Xinjiang 832003, China; 18799297836@163.com (X.L.); 18738595903@163.com (C.L.); e18899595697@163.com (Z.L.); 15739330255@163.com (R.Y.); 15136705752@163.com (Y.X.); 15509935295@163.com (R.Q.); mdzzhang@163.com (M.Z.); 15739333350@163.com (H.L.); 15609936261@163.com (L.L.); 2 College of Animal Science and Technology, Shihezi University, Xinjiang 832003, China

**Keywords:** circ-FoxO3, C2C12 myoblast cells, cell proliferation, cell differentiation, miRNA sponge

## Abstract

CircRNA is a type of closed circular non-coding RNA formed by reverse splicing and plays an important role in regulating the growth and development of plants and animals. To investigate the function of circ-FoxO3 in mouse myoblast cells’ (C2C12) differentiation and proliferation, we used RT-qPCR to detect the expression level of circ-FoxO3 in mouse myoblast cells at different densities and different differentiation stages, and the specific interference fragment was used to inhibit the expression level of circ-FoxO3 in myoblast cells to observe its effect on myoblast cells proliferation and differentiation. We found that the expression level of circ-FoxO3 in myoblast cells increased with the prolongation of myoblast cells differentiation time, and its expression level decreased with the proliferation of myoblast cells. At the same time, we found that the differentiation ability of the cells was significantly increased (*p* < 0.05), but the cell proliferation was unchanged (*p* > 0.05) after inhibiting the expression of circ-FoxO3 in myoblast cells. Combining the results of bioinformatics analysis and the dual luciferase reporter experiment, we found that circ-FoxO3 is a sponge of miR-138-5p, which regulates muscle differentiation. Our study shows that circ-FoxO3 can inhibit the differentiation of C2C12 myoblast cells and lay a scientific foundation for further study of skeletal muscle development at circRNA levels.

## 1. Introduction

Skeletal muscle is one of the most important components of animals (constitutes 40% to 50% of the animal body), is involved in exercise and energy metabolism, and is directly related to livestock growth and meat production [1,2]. The formation of skeletal muscle is influenced by many factors (genetic, environmental, nutrient, and disease) and is a very complex biological process regulated by genes, transcription factors, non-coding RNAs, and some signaling pathways [3,4,5,6,7,8]. Myogenesis is the process by which a somatic cell undergoes a series of proliferation, migration, and differentiation to form muscle tissue during development of the embryo [9,10]. Recent studies have shown that circular RNAs (circRNAs) have been identified as emerging non-coding RNAs during skeletal muscle development and play a crucial role in muscle development [11,12,13,14,15,16,17,18,19], but the specific functions in the proliferation and differentiation of myoblast cells are still unclear.

RETRACTED

CircRNAs are non-coding RNA molecules ubiquitous in eukaryotes that are formed by reverse splicing by non-canonical splicing [20]. Compared with traditional linear RNAs, circRNA molecules have a closed loop structure with no 5′ end cap and 3′ end poly(A) tail, which is resistant to the degradation of exonuclease RNaseR and, therefore, more stable than linear RNAs [21,22]. In 1976, the first circRNAs were discovered in the Sendai virus and plant-like viruses by Kolakofsky and Sanger [23,24], respectively, and only a few circRNAs were discovered until 1999 [25]. In the past few decades, circRNAs were considered to be a false shear product or transcriptional noise due to their low abundance and low functional potential [26], and their functions were unknown for a long time. In recent years, with the widespread use of RNA sequencing (RNA-seq) technology and the rapid development of biophysical technology, circRNAs can form by nonlinear alternative splicing or non-canonical exons [27,28]. Studies have shown that circRNA molecules contain an miRNA response element (MRE), which can act as competitive endogenous RNAs (ceRNAs) and bind with miRNAs to play the role of the miRNA sponge in the cell, in order to release the inhibitory effect of miRNA on target genes and regulate the expression level of target genes [29,30]. A well-known example is that ciRS-7 and Sry regulate the expression of downstream target genes by sponging miR-7 and miR-138, respectively [17,31]. Some studies have found that circRNAs are abundantly expressed in skeletal muscle tissue of many species to regulate myocyte development [12,17,32]. Circ-FoxO3 transcribes by the transcription factor FoxO3 gene, which mainly localizes in the cytoplasm and acts as a scaffold to bind to various RNA-binding proteins (RBPs) for forming stable complexes. Circ-FoxO3 forms an RNA-protein ternary complex with CDK2 and p21. This prevents CDK2 from interacting with cyclin A and E, which slows cell cycle progression [33]. For example, circ-FoxO3 interacts with ID-1, E2F1, and FAK, HIF1α, and the function of the latter are inhibited, which results in cell senescence [34]. The circBase search reveals that the isoform of circ-FoxO3 is highly conserved between the human and the mouse, which is located at chr6:108984657–108986092 in the human genome and chr10:41916271–41917707 in the mouse genome. The transcription gene FoxO3 belongs to the O subclass of the Forkhead family and consists of four members: FoxO1 (FKHR), FoxO3 (FKHRL1), FoxO4 (AFX), and FoxO6, which are characterized by a conserved DNA binding domain [2,35]. This family is present in all eukaryotes and is involved in many important biological processes such as substrate metabolism, protein turnover, cell survival, etc., and plays an important regulatory role in cell homeostasis [36,37]. The FoxO proteins are expressed in a variety of tissues, but their expression levels, functions, and targets are tissue-specific [36,38]. Among them, FoxO3 is mainly expressed in breast and leg muscles, and is involved in cell growth, development, and longevity. It is a crucial regulator of cell fate that controls proliferation, apoptosis, and differentiation and a key participant in the control of skeletal muscle protein turnover [36,39]. In a previous study, we found that the FoxO3 mRNA level was increased three-fold during myoblast cells to myotube transition [40]. FoxO3 as a candidate gene for chicken growth promotes myoblast cells proliferation and inhibits myotube differentiation in cells [41]. FoxO3 plays a key role in muscle atrophy and is essential for inducing skeletal muscle autophagy in vivo [42]. In summary, FoxO3 plays an important regulatory role in skeletal muscle tissue, but the specific mechanism of circ-FoxO3 in regulating the proliferation and differentiation of mouse myoblast cells (C2C12) is still unclear.

RETRACTED

In this case, we analyze the expression pattern of circ-FoxO3 and study its functions in proliferation and differentiation of mouse myoblast cells. Our study reveals that silencing circ-foxO3 promotes myoblast cells (C2C12) differentiation, which further reveals the regulation mechanism of muscle development and provides a new perspective for increasing muscle mass.

## 2. Materials and Methods

### 2.1. Ethics Statement

The experimental procedure in this study was performed in accordance with the requirements of the Statute on the Administration of Laboratory Animals and was approved by the Institutional Animal Care and Use Committee at Shihezi University (LS2018-108-01).

### 2.2. Tissue Sample Preparation

Three healthy, 4-week-old C57/BL6 mice were selected. We used isoflurane anesthesia and killed the mice with decapitation. The mice were carefully dissected in a sterile environment and their hearts, livers, spleens, lungs, kidneys, small intestines, and skeletal muscle tissues were collected. All samples were immediately frozen in liquid nitrogen and then stored at −80 °C until total RNAs extraction.

RETRACTED

### 2.3. RNA Extraction, cDNA Synthesis, and Quantitative Real-Time PCR (RT-qPCR)

We used Trizol (Invitrogen, Carlsbad, CA, USA) to extract total RNAs from seven tissue samples, according to the manufacturer’s instructions.The quality and purity of the RNAs were evaluated by 1.5% agarose gel electrophoresis, and then the concentration of RNAs were detected using a Nanodrop 2000 spectrophotometer (Thermo, Waltham, MA, USA). The PrimeScript RT kit (Takara, Dalian, China) was used to reverse transcribe total RNAs and synthesized first strand cDNA. The reaction system was 40:8 uL 5 × PrimeScript Buffer (for Real Time), 2 uL PrimeScript RT Enzyme Mix I, 2 uL Random 6 mers, 4 uL Total RNA, and 24 uL RNase Free ddH_2_O. The reaction was performed for 15 min at 37 °C and 5 s at 85 °C, according to the manufacturer’s instructions. Real-time fluorescence quantification (RT-qPCR) was performed using the LightCycler 480 system (Roche, Basel, Switzerland) with β-actin as an internal reference. The RT-qPCR was performed in a total volume of 20:10 μL of SYBR Green PCR Master Mix (Takara, Dalian, China), 0.5 uLof upstream primer and downstream primer, respectively, 1.0 μL of the cDNA template, and 8.0 μL of RNase-free water. All reactions were performed in triplicate and the specificity of the product was evaluated, according to the dissolution profile. The relative expression levels were calculated by 2-ΔΔCt. All primers were designed using Premier Primer 5.0 software and synthesized by RiboBio (Beijing, China). The detailed information is listed in Table 1.

### 2.4. Validation of Circ-FoxO3

Based on the NCBI reference sequence of FoxO3 (NCBI accession number: NM_019740.2) and circBase reference sequence of circ-FoxO3 (circBase ID: mmu_circ_0002207), a pair of back-to-back primers for specific amplification of the circ-FoxO3 gene were designed (Table 1). We extracted RNA from mouse skeletal muscle and reverse transcribed it into cDNA as a template. The circRNA junction site of circ-FoxO3 was amplified by polymerase chain reaction (PCR) using PrimerSTAR Max DNA Polymerase Mix (Takara, Dalian, China) to verify the presence of circ-FoxO3. The PCR product was detected by 1.5% agarose gel electrophoresis and DNA-seq. The DNA-seq result was analyzed using DNAMAN software (Lynnon Biosoft, Quebec, Canada).

### 2.5. Vector Construction

The precursor sequence of miRNAs (miR-96-5p (Hind III/BamH I), miR-138-5p (EcoR I/Xho I), miR-181a-5p (EcoR I/Xho I), miR-214-5p (Hind III/BamH I)) with flanking genomic sequence were amplified using Taq PCR MasterMix (Takara, Dalian, China). The PCR amplification product of miRNAs were inserted into vector of pcDNA3.1 (+) (Invitrogen, Carlsbad, CA, USA) by a restriction enzyme (Takara, Dalian, China) digestion and ligation to obtain an expression vector of miRNAs (pcD-miRNA). The full length of circ-FoxO3 was amplified and inserted into the 3′ end of the luciferase gene of the pMIR-Report Luciferase vector (Ambion, Shanghai, China) to generate wild pMIR-Report-circ-FoxO3-Wt plasmid (Spec I/Hind III). The overlapping extension PCR was used to amplify a completely mutated complementary sequence of the miR-138-5p seed sequence to generate the mutant pMIR-Report-circ-FoxO3-mut plasmid (Spe I/Hind III). All constructed vectors were verified by double enzyme digestion and DNA sequencing. Primer sequences were shown in Table 1.

RETRACTED

### 2.6. Cell Culture and Transfection

C2C12, which is an immortalized mouse myoblast cell line, was purchased from the cell bank of the Chinese Academy of Sciences. C2C12 is cultured in Dulbecco’s Modified Eagle Medium (DMEM) (Gibico, Grand Island, NY, USA) containing 10% fetal bovine serum (FBS) (Gibco, Grand Island, NY, USA) and 1% penicillin/streptomycin (Invitrogen, Carlsbad, CA, USA), and is cultured at 37 °C with a 5% CO_2_ humidified atmosphere. In order to induce the differentiation of C2C12, we replaced 10% FBS culture medium with 2% horse serum (HS) (Gibico, Grand Island, NY, USA) culture medium. We used liposomes 2000 (Invitrogen, Carlsbad, CA, USA) to transfect cells according to the manufacturer’s instructions. When the cell density reached about 80%, the culture medium was replaced with a Reduced Serum Medium (Gibico, Grand Island, NY, USA). After starvation treatment for 4 h, the cells were transfected with NC (siRNA mimic: 5′-UUCUCCGAACGUGUCACGUTT-3′) and siRNA (5′-GGGCAAAGCAGAACUCCAUTT-3′), respectively. After transfection for 6 h, the culture medium was changed into 10% FBS medium for subsequent experiments. NC and siRNA were synthesized by GenePharma Biotechnology (Shanghai, China).

### 2.7. Cell Proliferation and Differentiation Assay

We measured cell proliferation using the MTT Cell Proliferation Assay kit (Trevigen, Gaithersburg, Maryland, USA), according to the manufacturer’s instructions. After transfecting the siRNA for 24 h, the myoblast cells were resuspended and adjusted cell concentration to 6 × 10^4^/mL, and the cells were seeded into a 96-well plate at a density of 8000 cells/well in 100 μL culture medium. After incubating at 37 °C for 24 h and 48 h, we added a 20 μL MTT reagent (5 mg/mL) to each well, respectively. After incubating for 4 h, the liquid in each well was removed as much as possible. Additionally, 150 μL DMSO was added into each well and shaken at a low speed for 10 min on a shaker. Until the crystals at the bottom of the cell plate were completely dissolved, the absorbance value of each well was measured by a microplate reader at a wavelength of 570 nm. At the same time, zero adjustment holes (medium, MTT, dimethyl sulfoxide), control group (un-transfected myoblast cells, the same concentration of drug dissolution medium, culture solution, MTT, and dimethyl sulfoxide) were set, and was repeated 10 times per treatment. Excess holes were filled with sterile PBS.

RETRACTED

After transfecting the siRNA for 24 h, the growth medium was replaced with differentiation medium (DM, supplemented with 2% HS medium) (Gibico, Grand Island, NY, USA) and cultured for 3 days. The cells were collected and RNAs were extracted, respectively. The RT-qPCR was performed to detect the relative expression levels of the differentiation-related MyHC and MyoG genes. The day of shift to DM was indicated as 0 days of differentiation, and un-transfected myoblast cells as a control.

### 2.8. Dual Luciferase Assay

We transfected 800 ng microRNA expression vector, 400 ng firefly luciferase reporter plasmid pMIR-Report Luciferase (circRNA-Zfp609 wild type or mutant), and 80 ng Renilla luciferase reporter plasmid pRL-TK 293T cells in 12-well plates were transfected for 48 h. Co-transfected cells were lysed with 250 μL of cell lysis buffer. The Dual-GLO Luciferase Assay System kit (Promega, Madison, WI, USA) was employed to detect luminescent signals of firefly and Renilla Luciferase with a Fluorescence/Multi-Detection Microplate Reader (BioTek, Winooski, VT, USA), according to the manufacturer. Firefly luciferase activities were normalized to Renilla luminescence in each well.

### 2.9. Western Blotting

Cells from different treatment groups were collected and incubated on ice for 20 min using RIPA lysis buffer (Beyotime, Shanghai, China) containing 1 mM phenylmethanesulfonyl fluoroprotease inhibitor (PMSF) (Beyotime, Shanghai, China) to lyse the cells. The supernatant was then collected after centrifugation at 10,000× *g* and 4 °C for 10 min. The concentration of the extracted total protein was determined using a BCA protein concentration assay kit (Solarbio, Beijing, China). The expression of MyoG was detected by Simple WesternTM using a Proteinsimple Wes instrument (ProteinSimple, Santa Clara, CA, USA). The specific process was previously described [43]. The expression level of MyoG was detected by gray scale in the report. The primary and secondary antibodies used in the experiment were: anti-β-actin (1:2000, Abcam, Cambridge, MA, USA) and anti-myogenin (MyoG, 1:2000; Abcam, Cambridge, MA, USA) and goat anti-rabbit IgG (1:1000, Abcam, Cambridge, MA, USA).

RETRACTED

### 2.10. Statistical Analyses

ANOVA for P value calculations analyzed the results using SPSS v19.0 software (SPSS Inc, Chicago, IL, USA) and expressed as mean ± SD. There were at least three independent experiments with each treatment and *p* < 0.05 was statistically significant.

## 3. Results

### 3.1. Expression Pattern of Circ-FoxO3

The circ-FoxO3 was formed by the third exon of the FoxO3 gene on mouse chromosome 10. The circRNA junction site sequence of circ-FoxO3 was verified by RT-PCR (reverse transcription PCR) amplification using back-to-back specific primers (Figure 1A) and DNA-seq. Agarose gel electrophoresis detected RT-PCR products revealed a single band of expected size. At the same time, DNAMAN software analyzed the result of DNA-seq to confirm circ-FoxO3 (Figure 1B,C). Next, we isolated RNA from 7 different mouse tissues (Including heart, liver, spleen, lung, kidney, small intestine, and skeletal muscle) and reverse-transcribed into cDNA. RT-qPCR was used to detect the tissue specificity of circ-FoxO3. The results showed that circ-FoxO3 was expressed in various tissues, and its expression level was significantly different in different tissues. The expression level of circ-FoxO3 was highest in the heart and lowest in the kidney in all 7 mouse tissues examined (Figure 1D).

In order to further understand the function of circ-FoxO3, the process of C2C12 myoblast cells undergoes proliferation and differentiation. We initially tested changes in the expression level of circ-FoxO3 during the process of C2C12 myoblast cells proliferation and differentiation. First, we used RT-qPCR to detect the expression levels of circ-FoxO3 in C2C12 myoblast cells to the density of 50%, 80%, 100%, and more (>100%,over confluence). We found that the relative expression of circ-FoxO3 decreased with increasing C2C12 myoblast cells density (Figure 2A,B). Next, we examined the expression levels of circ-FoxO3 in C2C12 myoblast cells at different stages of differentiation: GM (proliferation phase), D1 (first day of differentiation), D3 (day 3 of differentiation), and D5 (day 5 of differentiation). The results showed that the expression level of the circ-FoxO3 gene was significantly up-regulated as the differentiation time progressed (Figure 2C,D).

### 3.2. Effect of Circ-FoxO3 on C2C12 Myoblast Cells Proliferation

To further investigate the effect of circ-FoxO3 on myoblast cells proliferation, we designed a methoxy-modified siRNA (2’Ome-modification) that specifically targets the circRNA junction site (the target site of siRNAs spans the junction site of circRNA) based on the circular structure of the circ-FoxO3 molecule. The siRNA interference efficiency was evaluated by transfecting into the C2C12 myoblast cells using liposome 2000 to detect the expression levels of the circ-FoxO3 gene and linear FoxO3 gene in the transfected C2C12 myoblast cells by RT-qPCR. Compared with the non-targeted control siRNA mimics, the expression level of circ-FoxO3 gene was significantly reduced by more than 95% (*p* < 0.05) and no significant effect on the expression level of linear FoxO3 gene (*p* > 0.05). This result indicates that our designed siRNAs can specifically interfere with the expression of circ-FoxO3 in C2C12 myoblast cells (Figure 3A). In addition, we determined the relative growth rate of myoblasts after siRNAs interference with circ-FoxO3 by the MTT assay, and the results show that interference with the expression of circ-FoxO3 in C2C12 myoblast cells have a slight inhibitory effect on cell proliferation, but the inhibitory effect was not significant (*p* < 0.05) (Figure 3B).

RETRACTED

### 3.3. Effect of Circ-FoxO3 on C2C12 Myoblast Cells Differentiation

The expression level of circ-FoxO3 grew with the increase of C2C12 myoblast cells differentiation time, so we hypothesized that circ-FoxO3 may play an important regulatory role in C2C12 myoblast cells’ differentiation. In order to understand the specific role of circ-FoxO3 in C2C12 myoblast cells’ differentiation, we transferred siRNAs that efficiently interfered with circ-FoxO3 expression into C2C12 myoblast cells to observe the effect of circ-FoxO3 on C2C12 myoblast cells differentiation. Compared with transfected non-targeted siRNA mimics, we found that the cell differentiation morphology of the experimental group was significantly different from that of the experimental group after three days of myoblast differentiation. The cell differentiation level of the experimental group was significantly higher than that of the control group (Figure 4A). Furthermore, RT-qPCR was used to analyze the expression levels of muscle differentiation-related genes (MyHC and MyoG) in the two groups. We found that the expression level of the MyHC gene in C2C12 myoblast cells was significantly increased when compared with the control group after interfering with the expression of circ-FoxO3 (*p* < 0.05), while the expression level of the MyoG gene did not change significantly (*p* > 0.05) (Figure 4B). At the same time, Western blotting results confirmed that the expression level of the MyoG gene in C2C12 myoblast cells was significantly increased after interfering with the expression of circ-FoxO3 (*p* < 0.05) (Figure 4C).

### 3.4. Prediction and Verification of the Interaction Between Circ-FoxO3 and miRNA

Numerous studies have shown that circRNA as a competitive endogenous RNA can function by acting as an miRNA sponge and regulating the expression of miRNAs and their target genes [44,45]. Therefore, in order to further understand the molecular mechanisms by which circ-FoxO3 plays a regulatory role in regulating muscle development, we used RNAhybrid and TatgetScan software to predict potential miRNA targets of circ-FoxO3. We found that several miRNAs associated with muscle development have potential targets for circ-FoxO3, including miR-96-5p, miR-138-5p, miR-181a-5p, and miR-214-5p (Figure 5A, Figures S1 and S2). Further studies using dual luciferase reporters revealed a significant decrease in luciferase activity when circ-FoxO3 was co-transfected with miR-138-5p (Figure 5B), so we choose miR-138-5p as a candidate for further studies.

RETRACTED

Based on two previously predicted potential sites of miR-138-5p that bind to circ-FoxO3, we designed two mutant primers to mutate all bases of the two binding sites. The electrophoresis results of PCR products showed a band of the expected size. The upstream and downstream sequences were spliced together by the overlap extension PCR method, and the electrophoresis results showed that the size of the band was consistent with the expectation (Figure S3). Next, we amplified and purified the mut-FoxO3-1/mut-FoxO3-2 gene and ligated it into the pMIR-Report luciferase vector (pMIR-Report-mut-circ-FoxO3-1, first site, pMIR-Report-mut-circ-FoxO3-2, second site). The constructed vector was digested with Spe I and Hind III, and a single band identical to the expected size was observed at 1436 bp (Figure 5C). This result indicated that the pMIR-Report luciferase vector was successfully constructed. The pcDNA3.1-miR-138-5p or pcDNA3.1(+) was co-transfected with pMIR-Report-mut-circ-FoxO3-1 or pMIR-Report-mut-circ-FoxO3-2 into 293T cells, respectively. There was no decrease in luciferase activity (all luciferase activities were homogenized by the Renilla luciferase activity) after co-transfection of pcDNA3.1-miR-138-5p and pMIR-Report-mut-circ-FoxO3-1 compared to the control (Figure 5D). These results indicate that miR-138-5p interacts with the predicted first target site in circ-FoxO3, which may be one of the pathways by which circ-FoxO3 regulates C2C12 myoblast cells’ differentiation even though further research is needed in the future.

## 4. Discussion

With the development of high-throughput sequencing, more and more circRNAs have been discovered in different cell types and tissues. As a new post-transcriptional regulator, circRNAs play an important biological role in many physiological and pathological processes and have become a hot spot in biological research [11,46,47,48]. However, currently, the regulation mechanism of circRNAs in skeletal muscle growth and development is still unclear. Therefore, studying the unique regulatory functions of circRNAs in skeletal muscle growth and development have become a hot topic at this stage.

RETRACTED

The FoxO transcription factor can be used as a general indicator of homeostasis, which regulates the cell cycle and controls individual cell integrity through a variety of different pathways. The current research indicates that the FoxO3 gene participates in the regulation of skeletal muscle development [49]. CircRNAs are more stable than linear mRNAs due to its covalently closed circular structure and long half-life [50]. Therefore, this study aimed to investigate the role of circ-FoxO3 in myoblast proliferation and differentiation. We examined the expression levels of circ-FoxO3 in different tissues of mice and found that its expression level in skeletal muscle is relatively low, which seems to indicate that the formation of circ-FoxO3 may be competitive with mRNA FoxO3. At the same time, we also examined the expression levels of circ-FoxO3 at different cell densities and differentiation stages. It was found that the expression level of circ-FoxO3 decreased with the increase of C2C12 myoblast cells density. However, the expression level of circ-FoxO3 was significantly increased with the degree of C2C12 myoblast cells differentiation. We found that, after silencing circ-FoxO3 by RNA interference, the differentiation of C2C12 myoblast cells were promoted, but the effect on proliferation were not significant. Further detection of differentiation marker genes in these C2C12 myoblast cells revealed that the expression levels of MyHC and MyoG were significantly increased. At the same time, the detection of MyoG gene expression levels at the protein level also confirmed this result. These results show that circ-FoxO3 can inhibit C2C12 myoblast cells’ differentiation but has no effect on C2C12 myoblast cells proliferation.

Studies have shown that circRNA act as an miRNA sponge to regulate post-transcriptional gene expression. For example, circFUT10 can absorb miR-133 to promote the myoblasts proliferation [51], Zfp609 circular RNA regulates myoblasts’ differentiation via sponge miR-194-5p [32], and circSVIL through sponge miR-203 promotes skeletal muscle cell proliferation and differentiation [52]. The above studies indicate that circRNA plays an important role in the regulation of cell function by regulating downstream target genes through sponge miRNA. We use biological informatics to predict miRNAs targeted by circ-FoxO3, and to detect predicted miRNAs (miR-96-5p, miR-138-5p, miR-181a-5p and miR-214-5p) associated with regulation of muscle growth and development using the dual luciferase reporter system. We found that the fluorescein reporter signal was significantly down-regulated when co-transfected with circ-FoxO3 and miR-138-5p, which indicated that miR-138-5p is a targeted miRNA of circ-FoxO3. At the same time, Xue et al. showed that miR-138 can affect the fibrosis of C2C12 cells by inhibiting the expression of target gene Smad4 [53]. To further understand the location of miR-138-5p targeting circ-FoxO3, we further mutated the two target sites of miR-138-5p in circ-FoxO3 predicted by bioinformatics and constructed luciferase reporter vectors, respectively. Compared to the control, there was no decrease in relative fluorescein activity when the first site was mutated, which suggests that miRNA-138-5p may be involved in the regulating mouse myoblast differentiation by targeting circ-FoxO3 at this site, even though further in-depth research is needed in the future.

RETRACTED

In summary, our study showed that the expression of circ-FoxO3 in different tissues of mice is tissue-specific and low in skeletal muscle. The expression of circ-FoxO3 decreased with increasing cell density and increased with increasing differentiation time. We have used RNA interference technology to show that circ-FoxO3 inhibits C2C12 myoblast cells’ differentiation. In addition, we validated the interaction of circ-FoxO3 with miR-138-5p using a dual luciferase reporter system and identified the target sites for interaction. This study provides a new perspective for circRNAs regulation of muscle development and provides new clues for the molecular basis of skeletal muscle development.

## Figures and Tables

**Figure 1:** Expression pattern of circ-FoxO3. (**A**) Divergent primers used in the amplification of circular junction. (**B**) RT-PCR verification of circ-FoxO3 junction site by reverse splicing. M is a marker (Takara, DL500: 500 bp, 400 bp, 300 bp, 200 bp, 150 bp, 100 bp, and 50 bp), and lane 1 is a negative control. (**C**) Validation of circ-FoxO3 head-to-tail junction sequence using DNA sequencing. (**D**) Differential expression of circ-FoxO3 in seven different tissues (heart, liver, spleen, lung, kidney, stomach, small intestine, and skeletal muscle) of a mouse. Expression levels in different tissues are normalized using the β-actin gene. All groups were performed with three biological replicates and all reactions were performed in triplicate. Error bars indicate ± SD.

**Figure 2:** Expression pattern of circ-FoxO3 during C2C12 myoblast cells’ proliferation and differentiation. (**A**) Cell morphology of C2C12 myoblast cells at different densities (50%, 80%, 100%, and over). (**B**) Detection of circ-FoxO3 expression levels in C2C12 myoblast cells of different densities (50%, 80%, 100%, and over) by RT-qPCR. We used the β-actin gene as an internal reference to normalize the relative expression levels of circ-foxO3 at different cell densities, and we used circ-foxO3 expression levels in samples with a cell density of 50% (set to 1) to quantify other samples. (**C**) Cell morphology of C2C12 myoblast cells at different differentiation times (GM, D1, D3, and D5). (**D**) Detection of circ-FoxO3 expression in C2C12 myoblast cells at different time points by RT-qPCR (GM, D1, D3, and D5). GM represents an undifferentiated state. D1, D3, and D5 represent the first day of differentiation, the third day of differentiation, and the fifth day of differentation, respectively. We used the β-actin gene as an internal reference to normalize the relative expression levels of circ-foxO3 at different differentiation times, and we used circ-foxO3 expression levels in GM samples (set to 1) to quantify other samples. All groups were performed with three biological replicates and all reactions were performed in triplicate. Error bars indicate ± SD, * *p* < 0.05, ** *p* < 0.01, and *** *p* < 0.001.

RETRACTED

**Figure 3:** Effect of circ-FoxO3 on C2C12 myoblast cells proliferation. (**A**) Verification of interference efficiency of circ-FoXO3 by siRNA. The expression levels of FoxO3 and circ-FoxO3 are normalized using the β-actin gene. NC is a siRNA mimic, and we used NC samples (set to 1) to quantify other samples. (**B**) Detection of the effect of circ-FoxO3 on C2C12 myoblast cells by the MTT assay. NC is a siRNA mimic, and we used NC samples (set to 1) to quantify other samples. All groups were performed with three biological replicates and all reactions were performed in triplicate. Error bars indicate ± SD and **** *p* < 0.0001.

**Figure 4:** Effect of circ-FoxO3 on C2C12 myoblast cells differentiation. (**A**) Differentiation morphology of C2C12 myoblast cells on day 3 after siRNA interference. NC is a siRNA mimic. (**B**) The expression of MyHC and MyoG in C2C12 myoblast cells on day 3 of differentiation after siRNA interference were detected by RT-qPCR. The expression levels of MyHC and MyoG are normalized using the β-actin gene. NC is un-transfected myoblast cells, and we used NC samples (set to 1) to quantify other samples. (**C**) The expression of MyoG in C2C12 myoblast cells on day 3 of differentiation after siRNA interference were detected by the Simple WesternTM assay. All groups were performed with three biological replicates and all reactions were performed in triplicate. Error bars indicate ± SD, * *p* < 0.05 and **** *p* < 0.0001.

RETRACTED

**Figure 5:** Interaction of circ-FoxO3 with miRNA. (**A**) Bioinformatics analysis predicts circ-FoxO3 potential miRNA target sites. (**B**) Identification of miRNA target sites of circ-FoxO3 by a dual luciferase reporter system. NC is a pcDNA3.1(+) empty plasmid, and we used NC samples (set to 1) to quantify other samples. (**C**) Double restriction enzyme digestion of a recombinant vector with miR-138-5p target site mutation. Lane 1 is a control plasmid. Lanes 2 and 3 are pMIR-Report-mut-circ-FoxO3-1 and pMIR-Report-mut-circ-FoxO3-2, respectively. M is a marker (Takara, DL10000: 10,000 bp, 7000 bp, 4000 bp, 2000 bp, 750 bp, 500 bp, and 250 bp). (**D**) The dual luciferase reporter system detects the fluorescence efficiency of co-transfected circ-FoxO3 mutants and pcDNA-miR-138-5p (co-transfected circ-FoxO3 mutants and pcDNA3.1(+) empty plasmid were used as a control group), and we used control group samples (set to 1) to quantify test group samples. All groups were performed with three biological replicates and all reactions were performed in triplicate. Error bars indicate ± SD, ** *p* < 0.01.

**Table 1:** The information of the primers used in this experiment.

Primer	Sequences	Tm/°C
circ-FoxO3-F	GGCCTCATCTCAAAGCTGG	58
circ-FoxO3-R	CTTGCCCGTGCCTTCATT	
linear-foxO3-F	CGCTGTGTGCCCTACTTCA	58
linear-foxO3-R	CTTGCCCGTGCCTTCATT	
FoxO3-F	CGGACTAGTAACTCCATCCGGCACAAC	64
FoxO3-R	CCCAAGCTTCTGCTTTGCCCATTTCC	
miR-214-5p-F	CCCAAGCTTCTGCATGAGGGCCAGTAAC	60
miR-214-5p-R	CGCGGATCCGCAGTGAATGTCGAGAGTGTG	
miR-181a-5p-F	CCCAAGCTTCTCCCTGTCTTTAACAGCCTG	62
miR-181a-5p-R	CGCGGATCCGCAGAAGTTAAACCGAGAAACG	
miR-96-5p-F	CCCAAGCTTTGGGGGGAGTAGGTTGTAG	64
miR-96-5p-R	CGCGGATCCAACAGGGCATCACAGAAGC	
miR-138-5p-F	CCGGAATTCTGCTGTGGACCTGGTATCTC	63
miR-138-5p-R	CCGCTCGAGCACAGGGGAGCAGTTCAA	
MyoG-F	CAATGCACTGGAGTTCGGT	58
MyoG-R	CTGGGAAGGCAACAGACAT	
MyHC-F	CGCAAGAATGTTCTCAGGCT	58
MyHC-R	GCCAGGTTGACATTGGATTG	
RT-mmu-β-actin-F	ATGGTGGGAATGGGTCAGA	58
RT-mmu-β-actin-R	TCAATGGGGTACTTCAGGGTC	
Mut- miR-138-5p-1-R1	AGATACAGCTGGCTGAGCCAAGGCTGCTGGAGT	64
Mut- miR-138-5p-1-F1	CTTGGCTCAGCCAGCTGTATCTAGCAGTCTCCCGCCAGCCAGTCTAT	
Mut- miR-138-5p-2-R2	CGTTGTAGAGCTCTTGGCGGTATATGGGAAGCTGG	64
Mut- miR-138-5p-2-F2	ATATACCGCCAAGAGCTCTACAACGGGCTCCCCAACCGGCTCCTTCA	

## Supplementary Materials

The following are available online at https://www.mdpi.com/2073-4409/8/6/616/s1. Figure S1: Several miRNAs associated with muscle development have potential targets for circ-FoxO3. Figure S2: miRNA vector construction. Figure S3: Construction of the circ-FoxO3 mutant. Supplementary Table S1: Amplification efficiency of RT-qPCR primers.
